# Factor Analysis and Mental Health Prevention of Employee Turnover under the Profit-Centered Development of Modern Service Industry

**DOI:** 10.1155/2022/3375386

**Published:** 2022-10-07

**Authors:** Youwen Zhong, Huifang Zhang, Xiaoling Wu

**Affiliations:** ^1^School of Economics and Finance, Xi'an Jiaotong University, Xi'an, Shaanxi, China; ^2^The Second Affiliated Hospital of Xi'an Jiaotong University, Xi'an, Shaanxi, China

## Abstract

Recently, the employee turnover rate of the modern service industry has continued to increase, leading to a decline in the service quality, customer turnover, and an increase in human costs. Meanwhile, fierce competition and enterprises' internal pressure have brought great psychological trauma to employees and affected their mental health. Understanding and finding out the factors that affect employees' resignations are the solutions to employees' mental health problems. The research innovation lies in building a relationship model between turnover intention, psychological contract, and job satisfaction; analyzing the influence mechanism and interaction of various variables in the model; and providing reference and thinking for the service industry to solve the problem of excessive turnover of employees. Besides, the questionnaire design and investigation are carried out, and 60 front-line employees of a service company are selected as the research objects. The results show that the overall internal consistency coefficient of SCL-90 is 0.96, and the overall consistency coefficient is directly proportional to the scale's reliability. The validity coefficient of SCL-90 is 0.79, which has good compatibility validity. Moreover, the correlation coefficient between the psychological contract and turnover intention is 0.621, and the Sig value is 0.00. The correlation coefficient between job satisfaction and turnover intention is −0.663, and the Sig value is 0.00. The psychological contract is positively correlated with turnover intention, and job satisfaction is negatively correlated with turnover intention. After the standard dance experiment, the *P* values of psychological indicators such as somatization, interpersonal relationship, depression, anxiety, and psychosis factors of employees in the control and experimental groups are all less than 0.05, indicating a significant correlation. Therefore, through 12 weeks of standard dance practice, all psychological indicators of the experimental group are significantly improved. However, the change results of the terror factor and paranoia factor are *P* > 0.05, showing no significant difference. After the standard dance experiment, there is a significant difference between the control and experimental groups in mental health factors, but no significant difference in terror and paranoia factors. This study has significant reference value for the prevention of employee turnover and mental health.

## 1. Introduction

The basic characteristics of the modern service industry are high human capital content, high added value, and high technology content. Human resources, technology, and knowledge have become the driving forces for its healthy development. Meanwhile, it is growing steadily in China's large and medium-sized cities and is expanding in-depth and breadth, increasing job opportunities [1]. At the same time, industrial agglomeration has also ushered in the era of modern service technology and knowledge sharing, raising employee possible turnover rate and intensifying the instability of the employment market. The competition among enterprises is in essence the competition of human resources, in which talents are the key. Thus, to ensure the normal and effective operation and development of enterprises, managers should focus on the introduction of excellent talents and the reduction of the turnover rate of talents. Today, talent flow has become a major social phenomenon [2]. By 2020, the turnover rate of the modern service industry has reached as high as 12.6%. Employee turnover rate is under heated discussion under many domestic online headhunters. Many scholars have also expressed their opinion about the cause of employee turnover and talent retention mechanisms. Besides, because of the fierce market competition among the service industry, employees often work under great psychological pressure, and some of them may suffer mental health problems. Attention to the sources of employees' psychological pressure and improvement on their mental health status has become the common goals of the government, enterprises, and employees [3].

This exploration is to study employee turnover from the perspective of the psychological contract and job satisfaction. The psychological contract emphasizes the mutual understanding of obligations in the employee-employer exchange relationship based on various forms of commitment, which is essentially the expectation of mutual responsibility. The psychological contract is often ignored because of its informality, fuzziness, and implicitness. It is not as binding as legal and economic contracts [4]. Changes in organizational structure and employment relationships can be reflected timely and accurately through psychological contracts. Job satisfaction is a key indicator reflecting employees' attitudes in the organization, and it is significantly related to some major behaviors of employees (including turnover rate), so it has attracted extensive research. Moreover, in order to alleviate employees' mental health problems and improve their mental health, it is essential to analyze the relationship between employees' turnover and international dance movement learning. As one of the sports dance items, standard dance is a normative and professional derivative of social dance. In the standard dance, the joints of the body actively participate in the music rhythm to exercise the body, cultivate the sentiment, and bring joy to the participants. It reveals that standard dance has positively reduced work pressure, improved negative emotions, and promoted interpersonal communication. Hence, according to the action recognition effect of standard ballroom dance, the mental health level of employees can be judged, and the turnover intention of employees can be further judged. Cheng et al. [5] studied the job burnout and satisfaction of employees. By analyzing the key moments of service interaction among front-line employees of hotels, considering workload and role pressure, they tried to solve the problem of employee burnout from the perspective of job design. The results show that higher job satisfaction greatly reduces the absence rate of employees and is a crucial factor to alleviate the turnover rate of employees. Mahajan et al. [6] studied the impact of customer satisfaction on employee performance in organizational work. The results show that employees are the most crucial part of the organization. Without employees, the company's organizational structure cannot exist. Hence, it is essential to focus on profits, analyze the factors that affect employees' turnover, and improve employees' job happiness and satisfaction.

Here, the employees in the modern service industry are sampled for QS (questionnaire survey), and their turnover factors and the prevention methods for their mental health problems are explored. The influencing relationship and mechanism between turnover intention and psychological contract and job satisfaction are analyzed and understood for the employees in the service industry. Then, from the perspective of the psychological contract, the influence mechanism of employee turnover intention in the service industry is studied, and solutions to reduce employee turnover rate are put forward, maintaining the stability and efficiency of the service industry. Additionally, the mental health problems of employees are treated through the experiment of standard dance exercise, and the related indexes of physical quality and mental state of employees before and after the experiment are compared and analyzed. The results provide scientific experimental data for the influence of standard dance exercise on the physical and mental health of employees so that employees can standardize and effectively carry out standard dance exercise, prevent and treat their mental health problems, and improve work efficiency, thereby enhancing the enterprise's efficiency and core competitiveness.

## 2. Methodology

### 2.1. Research Subjects

Through the screening of experimental objects, this exploration select 60 front-line employees of a service company as the research objects, including 30 male employees and 30 female employees. The nature of the company is catering service industry, and the specific responsibility of front-line employees is to serve customers and meet their specific needs when dining. Then, the QS about the factors affecting employees' intention to resign are conducted. The questionnaires are issued, recovered, and screened, and the final results are statistically analyzed. Subsequently, in the standard dance experiment, 60 employees are randomly divided into the experimental group and the control group. The QS is conducted by random sampling. First, 15 subjects are selected from 30 males. Then, 15 subjects are selected from 30 women, with 30 members in each group (15 males and 15 females). The control group is told to keep the original living habits, while the experimental group is arranged to perform standard dance exercises at customized class time and specific requirements. Before and after the experiment, the physical fitness index and mental health scale of the two groups of subjects are tested and analyzed.

### 2.2. QS Design

The research is carried out in the form of QS, and the questionnaire design is needed first. QS is divided into four parts:

The first part is the personal data scale, including the gender, age, education level, and marital status of the subjects.

The second part is the psychological contract scale. Based on the relevant literature and the psychological contract scale [7–9], the psychological contract scale has 20 items, including 4 items in the material incentive dimension, 9 items in the environmental incentive dimension, and 7 items in the growth opportunity dimension.  Table 1 shows the details.

The third part is the job satisfaction scale. Here, the psychological contract of employees in S company is taken as the research object. The job satisfaction scale is measured through comprehensive evaluation, and there is no measurement of one dimension. Four items are selected to measure job satisfaction based on the related scales developed by predecessors.  Table 2 presents the details.

The fourth part is the turnover intention scale. It is also measured by comprehensive evaluation. Six items are selected based on the turnover intention scale developed by predecessors to measure turnover intention.  Table 3 shows the details. After the completion of the questionnaire design, employees' turnover intention is investigated and data are collected by issuing questionnaires on the spot.

### 2.3. Szilagyi Turnover Process Model of Employee Turnover Intention

In the turnover process model, turnover intention factors include job nature, employee relations, organizational business, salary system, personal characteristics, and external job opportunities, including organizational factors, personal factors, and external factors. Therefore, the study of turnover intention must be comprehensive. Turnover intention is related to psychological contracts and job satisfaction. In addition to studying the antecedent variables of turnover intention, scholars and enterprises have put forward multiple valuable studies in reducing turnover intention, such as strengthening information management of human resources, providing an independent working environment, providing a flexible working system, paying attention to the growth and development of employees, paying attention to diversified value distribution, and cultivating learning organizations. Meanwhile, the Szilagyi model can provide evidence for the study of voluntary turnover. The core idea of this concept is to bring the education of employees into the salary system of enterprises.  Figure 1 displays the Szilagyi turnover process model.

Figure 1 shows that the nature of an employee's work and the organization's business will affect the employee's turnover intention. Besides, the salary system and external job opportunities will directly impact employees' turnover intention, and excessive employees' turnover intention will further lead to a decrease in business volume and affect the economic benefits of stores.  Figure 2 presents the comparison of mean values of each variable.

### 2.4. Prevention Methods of Mental Health Problems through the Standard Dance

#### 2.4.1. Questionnaire Method and Survey

Questionnaires are issued to 60 front-line employees (30 males and 30 females) of a service company. The basic information, health status, and daily exercise of the respondents are understood. Then, those who do not have regular exercise or serious physical diseases and have sufficient time and energy to participate in standard dance are determined as experimental subjects. Symptom Checklist 90 (SCL-90) has been proven to be highly reliable and effective by scholars and researchers. The overall internal consistency coefficient of SCL-90 is 0.96, and the overall consistency coefficient is directly proportional to the scale's reliability. The validity coefficient of SCL-90 is 0.79, which has good compatibility validity. Therefore, from the perspective of reliability and validity, the scale is suitable for studying employees' mental health [10, 11].

On April 12, 2020, 60 copies of the SCL-90 scale were distributed and recycled for the first time at the beginning of standard dance training. After 12 weeks of standard dance training, the SCL-90 scale was distributed to the subjects for the second time and was recovered and evaluated. Questionnaires were distributed and collected face to face. After that, the validity of the questionnaire was checked and evaluated.

#### 2.4.2. Evaluation of Employees' Mental Health Based on a Standard Dance

Through the experimental study, 60 employees are randomly divided into a control group and an experimental group, each with 30 members (15 males and 15 females). The control group will maintain their original living habits, while the experimental group will receive 12 weeks long standard dance training [12–15], twice a week and two hours each time.

Based on the national physical fitness measurement standards and evaluation system issued by the State Sports General Administration, the physical fitness indexes are determined: grip strength (strength quality index), sitting three-dimensional flexion (flexibility quality index), selection reaction time (sensitive quality index), and closed-eye single-legged standing (balance ability index). These four indexes of the members of two groups are measured both before and after the experiment to analyze the changes in the data. Based on the actual data, the accuracy of the analysis results of the data is ensured [16–18].

## 3. Research Results and Analysis

### 3.1. Statistical Analysis of Turnover Factors

To understand the status of the psychological contract [19], job satisfaction [20], and turnover intention [21] of sample employees in A company, the APAA19.0 is used for descriptive statistics, obtaining the following conclusions.

First, the mean employee psychological contract in A company is 3.284, at the upper-middle level. It shows that the psychological contract of employees in A enterprise is relatively high.

Second, the mean job satisfaction is 3.317, at the upper-middle level, indicating that the A company staff job satisfaction is relatively high.

Third, the mean turnover intention is 3.195, which is above the medium level, indicating that the turnover intention of employees in Company A is high. The standard deviation of turnover intention is too large, 0.8103, indicating that the deviation of turnover intention between employees is very large. The comparison of the mean values of the psychological contract, job satisfaction, and turnover intention is shown in Figure 2.

### 3.2. Discrimination Analysis of Turnover Factors

#### 3.2.1. Independent Sample T-Test of Gender

The gender of employees is a dual value control variable. Therefore, under the influence of the gender of different subject samples, the results of independent sample *t*-test analysis on the influence of gender on the average score can be obtained by analyzing the significance scores of the psychological contract, psychological dimension, job satisfaction, and turnover intention (Figure 3). Figure 3 shows that among the surveyed employees of company A, females' psychological contract and job satisfaction scores are higher than that of males, while males' turnover intention is higher than that of females.

#### 3.2.2. Independent Sample T-Test of Marriage

Employees' marital status is a double-value control variable, so an independent sample *t*-test can analyze the significance-discrimination of different marital status on psychological contract, psychological dimensions, job satisfaction, and turnover intention. For the sample employees of A company, the mean values of variables under different marital statuses are shown in Figure 4.

Figure 4 implies that of those surveyed employees of A company, unmarried groups show a higher score of the psychological contract, job satisfaction, and turnover intention over married groups. Particularly, the discrimination between the psychological contract of unmarried and married groups is the largest, followed by job satisfaction.

#### 3.2.3. Independent Sample T-Test of Age

To study the significance-discrimination of age on psychological contract, psychological dimensions, job satisfaction, and turnover intention, a sample *t*-test is conducted again. The means of variables of different ages for surveyed employees are shown in Figure 5.

Figure 5 suggests that of those surveyed employees, the 20–25-year-old group shows a lower psychological contract and job satisfaction than other age groups, while they have a significantly higher turnover intention than other age groups, indicating that in A company, young employees are the most unstable. The scores of the psychological contract, psychological dimensions, and job satisfaction of employees aged 31–35 years are higher than those of other age groups, but their turnover intention is significantly lower than that of other age groups, indicating that this age group is the most stable in A company, and they seldom quit.

#### 3.2.4. Independent Sample *T*-Test of Education

Here, the significance-discrimination is analyzed for education on psychological contract, psychological dimensions, job satisfaction, and turnover intention. The means of variables for different degrees of surveyed employees are shown in Figure 6.

Figure 6 implies that of those surveyed employees, the scores of psychological contract and job satisfaction get higher with the increase of education level, but for the psychological dimension, the discrimination between different education levels is small. Meanwhile, the highest scores of turnover intention go to employees with a college degree, followed by those with a bachelor's degree, and the employees with a master's degree or above are the most stable in the company.

### 3.3. Correlation Analysis between Turnover Intention and Psychological Contract and Job Satisfaction

Pearson correlation analysis of SPSS25.0 can analyze the correlation between turnover intention and employees' psychological contracts and job satisfaction.  Table 4 shows the results.

Table 4 reveals that the correlation coefficient between psychological contract and turnover intention is 0.621 and the Sig value is 0.00, indicating a significant positive correlation between psychological contract and turnover intention. The correlation coefficient between job satisfaction and turnover intention is −0.663, and the Sig value is 0.00, indicating a significant negative correlation between job satisfaction and turnover intention.

### 3.4. Regression Analysis of the Psychological Contract, Job Satisfaction, and Turnover Intention

#### 3.4.1. Regression Analysis of Psychological Contract and Turnover Intention

The regression analysis is carried out with psychological contract set as independent variable and turnover intention set as the dependent variable. The specific process is shown in Table 5.

Table 5 indicates that the regression coefficient *R*^2^ of psychological contract on turnover intention is 0.38, the adjusted regression coefficient *R*^2^ is 0.37, the statistics *F* = 40.175, and the Sig value is 0.00. It indicates that there is a linear regression relationship between psychological contract and turnover intention. The psychological contract has a significant predictive effect on turnover intention, and the psychological contract can explain 38% of the variation of turnover intention.

#### 3.4.2. Regression Analysis of Job Satisfaction and Turnover Intention

The regression analysis is carried out with job satisfaction set as the independent variable and turnover intention set as the dependent variable. The specific process is shown in Table 6.

Table 6 suggests that the regression coefficient *R*^2^ of job satisfaction to turnover intention is 0.436, the adjusted regression coefficient *R*^2^ is 0.43, the statistics *F* = 50.146, and the corresponding Sig value is 0.00. It proves that there is a linear regression relationship between job satisfaction and turnover intention. Job satisfaction has a significant predictive effect on turnover intention, and job satisfaction can explain 43.6% of the turnover intention variation.

### 3.5. Test Results of SCL-90 Scale after Standard Dance Exercise

To evaluate the mental health status of the subjects, it is essential to further judge and measure the emotional status of the subjects through the learning and understanding of the standard dance movements. The standard Waltz rhythm is 3/4 beat of strong, weak, and weak repetition, with a clear rhythm and smooth movements. Participants can relax and alleviate their negative emotions by performing a whole set of dance movements to the music. Tango is a 2/4 beat of the cycle of strength and weakness, with a strong rhythm and ups and downs, so participants often feel strong, stable, and confident. Collective classroom learning can stimulate participants to adapt to the environment and integrate into the crowd. The communication with teachers and students in and after class encourages participants to open up while familiarizing themselves with the environment. Mutual tolerance and encouragement are cultivated through practice. With the deepening of the dancing course, exercisers are organized to perform in the communities during the festivals, through which the performances gain much confidence and become cheerful in collective activities, and some even have expressed their wishes to show themselves. These results can positively adjust the participants' psychological states.  Table 7 shows the test results of each index of the SCL-90 psychological scale of the employees in the control group and the experimental group after the experiment. Of these, 10 indexes: somatization, compulsion, interpersonal relationship, depression, anxiety, hostility, terror, paranoia, psychosis, and others, are represented by capital letters A, B, C, D, E, F, G, H, I, and J, respectively.

Table 7 shows that after the experiment, the total score, total mean score, the total score of positive items, and the mean score of positive items in the experimental group are lower than those in the control group. Thus, after 12 weeks of standard dance exercise, the mental health status of 30 employees in the experimental group has improved, with specific differences in each index.

Figures 7 and 8 display that the mean score of the somatization factor in the experimental group after standard dance exercise is significantly lower than that in the control group, and the significance discrimination is large, indicating that the somatization status of the experimental group has been improved. The mean score of compulsion factor in the experimental group also has decreased significantly. Interpersonal relationship factor means also has reduced moderately. The mean depression factor of the experimental group is 1.18, showing a significant decrease. The mean score of anxiety factor in the control group is 1.45, which is significantly different from that in the experimental group, and the decrease in the experimental group is significant. Meanwhile, the mean score of the hostility factor has decreased. The discrimination between the mean scores of terror factors in the two groups is small. The mean score of the paranoia factor in the experimental group is 1.11, smaller than that in the control group. The mean of psychosis factors in the experimental group is also lower than that in the control group. The mean scores of other factors in the experimental group are also relatively low.

The comparison of experimental data shows that the *P* values of somatization, compulsion, interpersonal relationship, depression, anxiety, hostility, psychosis, and other factors in the control group and the experimental group are less than 0.05, indicating that there is significant discrimination. These eight psychological indexes of the experimental group employees are significantly improved through the 12-week standard dance exercise. However, the terror factor and paranoia factor show no significant discrimination, *P* > 0.05, so these two psychological indexes have been slightly improved through the 12-week standard dance exercise, and the impact is not significant.

### 3.6. Discussion

To sum up, employees' psychological contract status, job satisfaction, and turnover intention in service companies are analyzed. Through the independent sample test results of gender, marriage, age, education, and other factors, the correlation coefficient between psychological contract and turnover intention is 0.621, and the Sig value is 0.00, indicating a significant positive correlation between psychological contract and turnover intention. The correlation coefficient between job satisfaction and turnover intention is −0.663, and the Sig value is 0.00, indicating a significant negative correlation between job satisfaction and turnover intention. Besides, the regression coefficient *R* of job satisfaction to turnover intention is 0.436, and the adjusted regression coefficient *R*^2^ is 0.43. The statistic *F* = 50.146, and the corresponding Sig value is 0.00. It proves a linear regression relationship between job satisfaction and turnover intention. Janssen et al. [22] reviewed and studied the impact of employees' mental health. The diversity of employees' mental health and emotional changes were discussed based on mindfulness-based stress reduction. The results show that the increase of psychological stress, depression, anxiety, and occupational stress will affect employees' turnover intention. Dimoff and Kelloway [23] explored the influencing factors of workplace mental health training and leadership behavior. The results show that three hours of mental health training for employees may lead to significant behavioral changes three months after training. Moreno Fortes, Tian, and Huebner [24] conducted an experimental study on the overall mental health level of employees and explored the mediating and regulating role of burnout and optimism in explaining the empirical link. The results show that occupational stress and active mental health training can improve the level of mental health services. Therefore, in the management of modern service enterprises, it is necessary to pay attention to the psychological health level of employees, improve their job satisfaction, and further reduce their turnover rate.

## 4. Conclusion

The turnover factors of 60 employees of service industry company A are analyzed. The results show that the psychological contract and job satisfaction of employees in company A are in the middle level. Gender difference has no significant effect on psychological contract, psychological dimension, job satisfaction, and turnover intention. Marital status significantly impacts the environmental incentives and growth opportunities of employees' psychological contracts. Age difference has significant discrimination on job satisfaction and turnover intention. Education level has significant discrimination against job satisfaction of different educational levels. From the perspective of correlation analysis, the psychological contract has a significant positive correlation with turnover intention, and job satisfaction has a significant negative correlation with turnover intention. Besides, through 12 weeks of standard dance practice, the eight psychological indicators of the experimental group are significantly improved. However, there is no significant difference in the changes of the terror factor and paranoia factor (*P* > 0.05), so these two psychological indicators of the experimental group are only slightly improved by 12 weeks of standard dance exercise, and the impact is not significant. This exploration can provide a practical reference value for improving the mental health level of service employees. In terms of turnover intention, gender difference has no significant effect on psychological contract, psychological dimension, job satisfaction, and turnover intention. This exploration has practical guiding significance for analyzing the influencing factors of employee turnover.

The shortcomings are reflected from two aspects. Firstly, the sample scale has been confined to the A company, limiting the application value of the results. Secondly, the teachers of standard dance are not professional, so nonstandard dance movements may be taught during the teaching process. It is expected that in the follow-up research, the scope and size of the samples should be expanded to make the research results applicable in the modern service industry. Meanwhile, professional standard dance teachers will be invited to guide students' movements and further improve the mental health of employees.

## Figures and Tables

**Figure 1:** Szilagyi turnover process model.

**Figure 2:** Comparison of mean values of each variable.

**Figure 3:** Comparison of the mean values of different gender variables.

**Figure 4:** Comparison of the mean values of various variables in different marriage status.

**Figure 5:** Comparison of the mean values of different age variables.

**Figure 6:** Comparison of mean values of variables with different education.

**Figure 7:** Comparison of improvement of mental health indexes after the experiment.

**Figure 8:** Comparison of the total score and mean score after mental health experiment.

**Table 1:** Psychological contract scale.

Items	Question numbers	Questions	Options				
			Not at all affirmative.	Negative.	Not sure.	Affirmative.	Very affirmative.
Material incentive	1	Do you think your company pays wages in strict accordance with employees' job performance?					
	2	Do you think your company's salary is competitive in the same industry?					
	3	Do you think your company has a sound welfare system?					
	4	Do you think your company has a fair salary system?					

Environmental incentive	5	Do you think there is a friendly working environment?					
	6	Do you think the relationship between leaders and employees is harmonious?					
	7	Do you think the company's job security is very stable?					
	8	Do you think your colleagues are mutually helpful?					
	9	Do you think your leaders give you enough trust and respect?					
	10	Do you think your company cares about employees' life and state of mind?					
	11	Do you think your company has abundant work resources?					
	12	Do you think you can receive guidance during work?					
	13	Do you think your performance has gained approval?					

Growth opportunities	14	Do you think your work is challenging?					
	15	Do you think there is plenty of learning and training?					
	16	Do you think there are sufficient opportunities for promotion?					
	17	Do you think you have given many initiatives and work autonomy?					
	18	Do you think your talents can be fully exerted in your company?					
	19	Do you think your opinions are of any reference for company decisions?					
	20	Do you think you have a clear career objective in your company?					

**Table 2:** Job satisfaction scale.

Items	Question numbers	Questions	Options				
			Not at all affirmative.	Negative.	Not sure.	Affirmative.	Very affirmative.
Job satisfaction	21	Do you think you are satisfied with your current working environment and nature?					
	22	Do you think you are satisfied with the prospect in the company?					
	23	Do you think you have a good relationship with your colleagues, and you are mutually helpful?					
	24	Do you think you have a strong sense of belonging in your company?					

**Table 3:** Turnover intention scale.

Items	Questions number	Questions	Options				
			Not at all affirmative.	Negative.	Not sure.	Affirmative.	Very affirmative.
Turnover intention	25	Do you think you have the intention to leave your company?					
	26	Do you often enquire about employment information of other companies?					
	27	Are you planning to quit as soon as possible?					
	28	Do you think the current job is not suitable for you?					
	29	Do you think you will work for your company for a long time?					
	30	Do you think you will turn down offers from other companies?					

**Table 4:** Correlation analysis between turnover intention and psychological contract and job satisfaction.

Items		Psychological contract	Job satisfaction
Turnover intention	Pearson correlation efficiency	−.621^∗∗^	−.663^∗∗^
	Significance (two tailed)	.000	.000
	*N*	60	60

∗∗The correlation is significant at 0.01 level (two-tailed).

**Table 5:** Regression analysis of psychological contract on turnover intention.

Independent variable	Dependent variable	*r*	*R* ^2^	Adjusted *R*^2^	*F*	Sig
Psychological contract	Turnover intention	−0.621^a^	0.380	0.370	40.175	0.000^a^

^a^Indicates that the significance level of data has passed the test, which has explanatory significance for the experimental results.

**Table 6:** Regression analysis of job satisfaction on turnover intention.

Independent variable	Dependent variable	*r*	*R* ^2^	Adjusted *R*^2^	*F*	Sig
Job satisfaction	Turnover intention	−0.663^a^	0.436	0.430	50.146	0.000^a^

^a^Indicates that the significance level of data has passed the test, which has explanatory significance for the experimental results.

**Table 7:** Index score table of the control group and experimental group after experiment.

Indexes	Letter	Control group	Experimental group	*P*-value
Somatization	A	1.56 ± 0.35	1.31 ± 0.27	<0.05
Complusion	B	1.34 ± 0.4	1.15 ± 0.26	<0.05
Interpersonal relation	C	1.38 ± 0.31	1.21 ± 0.19	<0.05
Depression	D	1.34 ± 0.34	1.18 ± 0.24	<0.05
Anxiety	E	1.45 ± 0.32	1.24 ± 0.29	<0.05
Hostility	F	1.37 ± 0.39	1.17 ± 0.17	<0.05
Terror	G	1.23 ± 0.25	1.08 ± 0.21	
Paranoia	H	1.18 ± 0.26	1.11 ± 0.17	
Psychosis	I	1.26 ± 0.21	1.16 ± 0.13	<0.05
Other	J	1.48 ± 0.32	1.21 ± 0.19	<0.05
Total score		121.34 ± 20.87	105.79 ± 13.68	
Total mean score		1.23 ± 0.28	1.02 ± 0.19	
Positive items		22.81 ± 12.67	16.79 ± 10.13	
Mean score of positive items		2.53 ± 0.41	2.13 ± 0.24	

## Data Availability

The raw data supporting the conclusions of this article will be made available by the authors, without undue reservation. The data used to support the findings of this study are included within the article.
